This article has been retracted.

# Clinical Characteristics and Treatment of Adult Idiopathic Carpal Tunnel Syndrome Accompanied with Trigger Digit

**DOI:** 10.1155/2022/8104345

**Published:** 2022-10-11

**Authors:** Jinjiong Hong, Xiaofeng Wang, Jianbo Xue, Jimin Li, Minghua Zhang, Weisheng Mao

**Affiliations:** Department of Hand Surgery, Department of Plastic Reconstructive Surgery, Ningbo No. 6 Hospital, China

## Abstract

**Purpose:**

To investigate the clinical characteristics and treatment of adult idiopathic carpal tunnel syndrome (CTS) accompanied with trigger digit.

**Materials and Methods:**

A retrospective analysis was performed on a total of 74 patients with adult idiopathic CTS accompanied with trigger digit admitted to and treated at the Hand Surgery Department of Ningbo No. 6 Hospital from January 1, 2017 to December 31, 2019. Data on patients' gender, age, occupation, course of the disease, menstruation, surgeries, examination-related information, complications, treatment methods, and prognoses during follow-up were recorded and subsequently used to analyze the pathogeneses, clinical characteristics, and treatment.

**Results:**

A total of 74 patients (72 females and 2 males) were included. Among female patients, 51 were postmenopausal and 18 were non-postmenopausal. There were 101 fingers with trigger digit, including 14 patients with trigger digit in both hands, and 115 wrists affected by the CTS. The average course of CTS was 34.5 ± 49.3 months, and that of trigger digit was 10.5 ± 22.4 months. Seventy had both trigger digit and CTS in one hand, while among patients with both hands involved, only 4 had trigger digit or CTS in one hand. Eighty-nine fingers underwent A1 pulley release, and 104 hands underwent carpal tunnel surgery, with steroids being injected under the adventitia of the median nerve during the surgery. All patients who underwent surgeries had I/A-healed incisions, and 14 of them had obvious synovial hyperplasia observed in the carpal tunnel and flexor tendon sheath during surgeries. Follow-up visits, which lasted 3 to 35 months, had an average duration of 1.34 years and included 72 patients. In 63 patients (63/72), the syndrome of tenosynovitis and numbness disappeared and normal hand functions were restored; in 6 patients, the numbness in hands greatly improved and normal hand functions were almost completely restored, while no improvement in numbness of hands and limited hand functions were still observed in 3 patients.

**Conclusion:**

CTS accompanied with trigger digit was more common in postmenopausal females, and the course of CTS was longer than that of trigger digit. CTS and trigger digit were more likely to simultaneously occur in the same hand, while some patients might not have obvious synovial hyperplasia in the carpal tunnel. Surgeries were effective in severe cases.

## 1. Introduction

Idiopathic carpal tunnel syndrome (CTS) and stenosing tenosynovitis, also known as trigger digit (TD), are common diseases treated at hand surgery departments [1–3]. Existing studies have suggested that multiple factors, such as age, gender, diabetes, perimenopause, pregnancy, rheumatoid arthritis, and other inflammatory arthritis and engagement in assembly line works, may increase the risk of CTS [4]. Some studies suggested that CTS accompanied with TD may occur in the same hand, successively or simultaneously [5, 6]. Yet, CTS with TD simultaneously is less common [7], and factors related to the risk of the onset of CTS with TD and its treatment have not yet been reported. The aim of this study was to investigate patients' clinical characteristics and treatment.

## 2. Materials and Methods

A retrospective analysis was performed on patients with CTS admitted to and treated at the Hand Surgery Department of Ningbo No. 6 Hospital from January 1, 2017 to December 31, 2019. In this study, adults with symptoms of CTS and TD were enrolled. The criteria for exclusion were malignancy, less than 20 years old, pregnancy, a history of forearm and hand trauma, CTS induced by tophus, tumor lesion, or wrist infection (e.g., nonmycobacterium tuberculosis infection), traumatic peripheral nerve injury and central nervous system diseases, and recurrent CTS. Patients with gout-induced stenosing tenosynovitis, tuberculous tenosynovitis, infective tenosynovitis, and other secondary tenosynovitis were also excluded. All of the patients were admitted to the hospital after invalid conservative treatment since the onset of the disease. The study was approved by the ethics committee of the Ningbo No.6 Hospital in Zhejiang (China). All patients signed informed consents at admission.

### 2.1. Statistical Analysis

SPSS software for Windows 13.0 (SPSS Inc., Chicago) was used to analyze all data. A *P* value of <0.05 was considered to be statistically significant. Measurement data were expressed as mean ± standard deviation (SD), and the two-independent-samples *t*-test was used for data analysis.

## 3. Results

Eventually, 74 patients were included in the study, including 72 females aged 40 to 71 years old (average age of 53.9 ± 6.7 years) and only 2 males aged 32 and 68 years old, respectively (Figure 1).

Among female participants, there were 51 postmenopausal, 18 non-postmenopausal, and 3 women who underwent hysterectomy before menopause. In terms of occupation, there were 29 operating workers, 25 housekeeping workers, 18 farmers, 1 office worker, and 1 freelancer. The course of the disease ranged from 6 months to 15 years, with an average CTS course of 34.5 months and an average TD course of 10.5 months. One of the patients suffered from chronic gastric ulcer, 3 had hysterectomy, 1 had thyroidectomy, 1 had arrhythmia, 1 had oophorocystectomy, 1 had hyperthyroidism, 5 had diabetes, and 14 had hypertension.

### 3.1. Disease Status and Examinations

In total, there were 101 fingers (including 46 on the left hand and 55 on the right hand) with TD, including 52 thumbs, 7 index fingers, 29 middle fingers, 11 ring fingers, and 2 little fingers. Based on the classification described by Lim et al. [8], the study included 3 Grade I (3%), 9 Grade II (9%), 78 Grade III (77%), and 11 Grade IV (11%) trigger digits.

Moreover, a total of 115 hands involved carpal tunnel presentation, with 41 patients having CTS in both wrists, 11 patients having CTS in the left wrist, and 22 patients having CTS in the right wrist. According to the electrophysiological grading of severity of CTS proposed by Padua et al. [9], 22 carpal tunnels were graded as mild (MILD), 43 as moderate (MOD), 47 as severe (SEV), and 3 as extremely severe (EXT) (Table 1 and Figure 2). If a patient had both TD and CTS in one hand, he/she was classified as an ipsilateral patient, regardless if he/she had TD and/or CTS in the other hand. If a patient had only TD or CTS in either hand, he/she was classified as a nonipsilateral patient. Finally, there were 70 ipsilateral patients and 4 nonipsilateral patients. Specifically, there were 12 ipsilateral patients with both hands involved and 58 ipsilateral patients with only one hand involved (including 24 with the left hand involved and 34 with the right hand involved).

All of the 74 patients underwent preoperative X-ray examination and electrophysiological examination of the median nerve, while some were selectively given cervical MRI, wrist MRI, and diagnostic ultrasonography. The X-ray examination, which was used to rule out the possibility of median nerve compression induced by malunion of an old fracture of the distal radius with lunate dislocation, confirmed that none of the patients had signs of fracture-induced dislocation, bone tumor, or bone erosion.

Patients with stenosing tenosynovitis and idiopathic CTS accounted for 8.4% of all patients with CTS who were admitted to the hospital (74/884). Among female patients, 51 were postmenopausal aged 44 to 71 years old (average age of 56.6 ± 5.8 years), with the average age of menopause being 49.5 ± 3.0 years old, including 1 patient who underwent a hysterectomy after menopause. The menopause in these women started at the average age of 49.5 ± 3.0 years, with the duration of menopause ranging from 0.5 to 20 years (average of 7.1 ± 5.7 years). There were 18 non-postmenopausal female patients aged 40 to 53 years old (average age 47.1 ± 3.7 years). The ages of non-postmenopausal female patients and postmenopausal female patients approximately conformed to the normal distribution; thus, two-independent-samples *t*-test was used to analyze them with *P* value of <0.05.

Among the 74 patients, there were 101 fingers with TD, including 52 thumbs, 7 index fingers, 29 middle fingers, 11 ring fingers, and 2 little fingers, with the thumbs accounting for 51.5% (52/101). Of all patients, 52 patients had one finger with TD, accounting for 70.3% (52/74), and 22 had multiple fingers with TD, accounting for 29.7% (22/74); 14 patients had both hands with TD, accounting for 19% (14/74), including 9 patients with both thumbs involved, accounting for 64% (9/14), and 2 patients having multiple (two or more) fingers on both hands involved. Among the 74 patients, CTS was found in 115 hands, with those severely and extremely severely involved, accounting for 43.5% of the total (50/115), and those with CTS in both hands, accounting for 55.4% of all patients (41/74), including 13 patients diagnosed with severe and 1 patient diagnosed with extremely severely CTS, accounting for 34.1% of all patients having CTS in both hands (14/41). Of all patients, 94.6% (70/74) had both TD and CTS in one hand.

The average course of CTS was significantly longer compared to the TD course, lasting 34.5 ± 49.3 months and 10.5 ± 22.4 months, respectively (*P* < 0.01). Forty-six patients had a longer course of CTS than TD, including 2 patients who underwent blocking of the diseased wrist and 2 patients who underwent blocking of the diseased finger during the course of the disease. The average course of CTS in these 4 patients was 50.0 ± 56.0 months, and that of TD in patients was 6.5 ± 11.9 months (*P* < 0.01). Comparatively, 11 patients had a longer course of TD than CTS, including 2 patients who underwent intrathecal injection of steroids during the course. Furthermore, 17 patients simultaneously had CTS and TD, with an average course of disease of 7.2 ± 9.2 months.

### 3.2. Treatment Methods

All surgeries were performed by senior hand surgeons. According to the severity of stenosing tenosynovitis, 12 fingers were given conservative treatment: 6 fingers of grade I and grade II patients who were given external application of Voltaren emulsion and local immobilization, and 6 fingers that were treated with intrathecal injection of steroids.

Eighty-nine fingers of grade III and grade IV patients were treated with A1 pulley release. In one patient with right thumb TD and moderate right CTS with the course of TD lasting 6 months who was treated with A1 pulley release of the right thumb and conventional open carpal tunnel release surgery, a long segment of large partial-rupture and adhesion in the flexor longus tendon was observed during the surgery, after which the patient was given a graft of palmaris longus.

Three wrists were treated with simplex intrainjection of steroids, 8 wrists with conservative immobilization treatment for the carpal tunnel, and surgery and injection of steroids under the neural adventitia were used to treat the carpal tunnel in 104 wrists, including endoscopic carpal tunnel release (ECTR) performed in 42 wrists, miniopen carpal tunnel release (MOCRT) performed in 39 wrists, mini-incision OCTR performed in 15 wrists, and conventional large OCTR performed in 8 wrists [10]. One patient who had severe CTS in the right wrist and tenosynovitis in the 2nd to 4th fingers on the right hand with the course of the disease lasting over about 15 years received A1 pulley release, OCTR, and palmaris longus tendon transfer for improving thumb function. Fourteen patients in the study had obvious synovial hyperplasia observed in the carpal tunnel with or without flexor tendon sheath during surgery, in whom the synovium was removed and sent for pathological test, which suggested fibrous synovial tissue hyperplasia. Clinical results at the final follow-up were evaluated according to the criteria of Kelly et al. [11]

TD symptoms significantly improved in all patients; numbness was significantly alleviated in 66 patients and 107 hands, while 8 patients with 8 hands, of which 3 hands were graded extremely severe and 5 were graded severe according to electrophysiological grading of severity before surgery, showed no significant alleviation of numbness. On Day 1 after surgery, TD symptoms and numbness did not aggravate in any of the patients. All incisions in the patients' given surgery were I/A-healed. Follow-up visits were completed in 72 patients and lasted 3 to 35 months, with an average duration of 1.34 years. According to the results at the final follow-up, sixty-three patients (63/72) experienced tenosynovitis; the numbness disappeared, and normal hand functions were restored; numbness was greatly improved, and normal hand function was almost completely restored in 6 patients, while 3 patients showed no improvement in numbness of hands and continued to have limited hand function. Using Kelly's criteria was excellent in 63 patients (87.5%), good in 6 patients (8.3%), and poor in 3 patients (4.2%).

## 4. Discussion

### 4.1. Factors Related to the Pathogenesis of Adult Stenosing Tenosynovitis with CTS

Previous studies have shown that women are more prone to CTS and that idiopathic CTS is more often seen in women than in men, while TD is the most often seen in women aged 40 to 60 years old [1]. Idiopathic CTS shows a female predominance and epidemiologic studies have shown that postmenopausal status or oophorectomy, which both represent fluctuations in estrogen level, is associated with idiopathic CTS [11]. According to McKinlay et al., women on average go through perimenopause at 47 years of age and, with the continuous depletion of ovarian follicles in middle age, they eventually experience changes in menstrual patterns and fluctuations in hormonal levels. Postmenopausal women are more prone to idiopathic CTS, which is related to steroid hormones, especially estrogens [13]. According to Kim et al. [12], marked increases in the expressions of estrogen receptor-*α* and estrogen receptor-*β* were found in the tenosynovial tissues of postmenopausal idiopathic CTS patients. Kaplan et al. believed that hypoestrogenic might affect the median nerve or other carpal tunnel structures, thus resulting in CTS [15]. In our study, the fact that there were more postmenopausal women suggested that postmenopause was the pathogenesis of stenosing tenosynovitis with CTS, although there was a lack of convincing evidence for the correlation between the onset of tenosynovitis and estrogen fluctuation in postmenopausal women. It might also be intriguing to investigate into the incidence of CST and TD in other complicated conditions [16–21].

According to Vance et al., around 1.5% to 20% of diabetic patients have secondary TD [22]. Ashour et al. [23] pointed out that the lifetime incidence of TD in the healthy population was 2.6%, and that in the diabetes population, it was as high as 16.5%. In a prospective study that included 160 patients with stenosing tenosynovitis, 38 had diabetes, accounting for 23.7% [24], while in this retrospective study, 5 patients with CTS and TD also had diabetes, accounting for only 7% of patients. There still lacks evidence for the significant correlation between diabetes and the onset of CTS with TD.

Adult TD may occur in one or more fingers on one or both hands and more often in the thumbs, middle fingers, and ring fingers. A previous study found that patients having TD in both hands accounted for 19% (14/74) of the total, where 64% (9/14) had both thumbs involved. Also, those having CTS in both hands accounted for 55.4% (41/74), where those having SEV and EXT accounted for 34.1% (14/41). Some observational reports suggested that TD was related to occupation or frequent hand activities. Nonetheless, this is still being disputed as some scholars believe that repeated hand working, especially repeated pinching and gripping at the flexor position and repeated flexing and stretching of the tendons of hands, may result in CTS induced by synovial hyperplasia of flexor tendons [25]. Previous studies using MRI provided strong arguments that idiopathic CTS development was closely related to the abnormality of synovial tissues in the carpal tunnel [26]. Ten et al. [3] suggested that CTS might result from tenosynovitis without significant clinical symptoms, which could be detected by ultrasonography. They also believed that synovitis symptoms observed in surgeries and ultrasonography were usually reactive changes responding to mechanical stress or pressure in the carpal tunnel. Our results showed that operating workers and long-term housekeeping workers accounted for 73.0% of all patients (54/74), and the involvement of both hands was more common in such patients. This suggested that TD with CTS was greatly related to occupation or frequent hand activities. Especially after the disease involved the wrist or thumb on one hand, the activities of the other hand increased as compensation, eventually resulting in the involvement of both hands.

### 4.2. Analysis of Characteristics and Causes of Adult Stenosing Tenosynovitis with CTS

TD is one of the most common causes of hand pain in adults and often the leading cause of frequent visits to the hospital. CTS patients develop numbness and tingling in fingers at the early stage of the disease, which is aggravated as the disease progresses, especially at night, thus affecting sleep. Some patients may visit the hospital only for numbness of the middle finger. With the disease's progression, patients develop atrophy of the thenar muscle and lack the strength of the thumb against the palm. Some patients may also visit the hospital only for atrophy of the thenar muscle and feel no sensory disturbance. Our results showed the course of TD in such patients was similar to that in patients having CTS and TD at the same time. Therefore, it is possible that patients with a longer course of CTS than TD did not visit the hospital in time for initial symptoms of CTS, while patients having CTS and TD at the same time visited the hospital more timely. The tolerance and repeatability of the initial symptoms of CTS might explain the delayed visit to the hospital in the majority of patients at the early stage of the disease. Patients with early CTS visited the hospital only after they had TD that caused hand pain.

The flexor tendon moves from the forearm to the far side through the carpal tunnel and enters the flexor sheath pulley system of fingers so that it can glide freely in this bone-fiber channel. In most patients with TD, the compression occurs at the A1 pulley. According to a previous study, the main histopathological change in patients with TD was the metaplasia of fibrous cartilage in the ligamentum layer of tendon sheath at A1 pulley, accompanied by secondary reduction of the cross-sectional area of the fibrous bone tunnel [27]. In the present study, 14 patients had obvious synovial hyperplasia in the carpal tunnel, and TD with CTS more often occurred in one hand, accounting for 94.6% of the total (70/74). This could be explained by the cooccurrence of tenosynovitis in the tendon sheath and carpal tunnel, which might be the result of the anatomical features of the flexor tendon gliding in the two-way (carpal tunnel-tendon sheath) tandem channel. CTS and TD occurred in different hands in 4 patients in the present study, which might be related to systemic factors such as gender, age, and hormonal levels. Also, CTS and TD might involve both hands in some cases due to being independent of each other.

### 4.3. Treatment for CTS with TD

The treatment for idiopathic CTS with stenosing tenosynovitis is basically the same as that used for individual treatment of these conditions, and it includes conservative treatment and surgical treatment. It is currently believed that surgical treatment for CTS is more effective, especially in the long run than splintage and other conservative treatments [28]. Carpal tunnel release (CTR) that cuts the transverse carpal ligament (TCL) is considered the most reliable method to improve the symptoms. Surgical treatment of CTS, which depends on surgical vision and how surgeons cut the TCL, is divided into the conventional open carpal tunnel release surgery, mini-incision carpal tunnel incision, MOCTR, double-incision carpal tunnel incision, and endoscopic surgery [29]. The use of the surgical method is mostly at the personal discretion of the surgeon. Patients with obvious synovial hyperplasia may be treated with synovial dissection around the flexor tendon after CTR. Our data showed that surgical treatment had satisfactory results, although some patients had commemorative irreversible neurological dysfunction due to the long course of CTS and delayed treatment. However, there was no evidence for the necessity of synovial dissection after incision of the A1 pulley and the transverse carpal ligament. Moreover, 14 patients with CTS and TD had obvious synovial hyperplasia observed in the carpal tunnel during surgeries, accounting for 19.0% of all patients. According to Ten et al., the clinical efficacy of carpal tunnel incision might be better when tenosynovitis is suggested in ultrasonography, and the carpal tunnel is subject to excessive internal pressure [3]. However, cutting the transverse carpal ligament may cause surgical risks and complications, such as injuries to the palmar cutaneous branch, the thenar branch of the median nerve, the superficial palmar arch or flexor tendon, and secondary stenosing tenosynovitis, in either the conventional CTR or endoscopic CTR [6]. Studies on synovial specimens from patients with idiopathic CTS showed that only 10% had inflammatory changes [30], and the majority showed edema or fibrosis. Different from patients with CTS induced by nonmycobacterium tuberculosis infection, some patients with CTS and TD did not have obvious abnormal synovial hyperplasia in the tendon sheath or carpal canal, which might be due to other possible unknown diseases or pathogenic factors in such patients that should be addressed by further studies. The treatment for idiopathic CTS with TD with obvious synovial hyperplasia in the carpal tunnel by removing proliferated synovial tissues and retaining the transverse carpal ligament after complete laboratory examinations needs to be further explored and studied.

## 5. Conclusion

In summary, we found that CTS accompanied with trigger digit was more common in postmenopausal females, and the course of CTS was longer than that of trigger digit. CTS and trigger digit were more likely to simultaneously occur in the same hand, while some patients might not have obvious synovial hyperplasia in the carpal tunnel. Surgeries were effective in severe cases.

## Figures and Tables

**Figure 1:** Flow chart of patients in this study.

**Figure 2:** Distribution of TDs.

**Table 1:** Characteristics and electrophysiological grading of severity of CTS of the patients.

Characteristics	Type	Number of cases (%)
Gender	Female/male	72/2 (97.3/2.7)
Menstruation	Postmenopausal females/non-postmenopausal females/others	51/18/3 (70.8/25/4.2)
Average age (year)	Postmenopausal females	56.6 ± 5.8
The average course of CTS (month)		34.5 ± 49.3
The average course of TD (month)		10.5 ± 22.4
Electrophysiological grading of severity of CTS	Severe (SEV)	47 (40.9)
	Moderate (MOD)	43 (37.4)
	Mild (MILD)	22 (19.1)
	Extremely severe (EXT)	3 (2.6)

## Data Availability

The data used to support the findings of this study are available from the corresponding author upon request.
